# Modeling Intention-Based Critical Determinants of E-Commerce Utilization: Emerging Business Models and Transformation in the Digital World

**DOI:** 10.3389/fpsyg.2022.889147

**Published:** 2022-08-10

**Authors:** Tianjie Tong, Yuyu Xiong

**Affiliations:** ^1^Graduate School of Business, SEGI University, Petaling Jaya, Malaysia; ^2^Postgraduate Department, Henan Agricultural University, Zhengzhou, China

**Keywords:** intention, critical factors, consumers, E-commerce, China

## Abstract

Companies in the world today understand that keeping users in touch is essential to enhancing their trust. The primary objective of this study was to determine the intention-based critical determinants of E-commerce utilization in China from the end users’ perspective. We developed a framework that identifies the factors that influence E-commerce utilization in China. Besides, we introduced observational research (data analysis) conducted in a real-world E-commerce sense. Results are based on a sample of 400 respondents by employing a comprehensive questionnaire survey. The structural equation modeling (SEM) and the partial least squares (PLS) regression approach was used to analyze the data. Study results show that perceived usefulness, perceived ease of use, reputation, trust in vendors, and purchase frequency significantly influence consumers’ intention to use E-commerce systems. Research outcomes emphasize transforming social norms, raising consumers’ awareness, redesigning policy frameworks, and highlighting the paybacks that E-commerce offers through integrative and consistent efforts.

## Introduction

Global E-commerce purchasing is about to hit US$4.2 trillion, and recent data show almost 27% growth in the E-commerce business (Uzir et al., 2021). According to statistics from the China Internet Network Information Center, the total number of online shopping users in China in June 2019 was 639 million, accounting for 74.8% of the total number of Internet users in the country, an increase of 28.71 million from the end of 2018. This trend of growth in E-commerce businesses is due to excessive use of the Internet and mobiles. E-commerce is altering the mechanisms by which businesses design, manufacture, and give their goods and services, as well as the number of customers who trust businesses. According to Eurostat reports, in 2011, a 65% increase in the number of businesses with an E-commerce thread occurred, and roughly half of such big businesses at the European commission already have it. According to Yang et al. (2021), offerings focused purely on responsible action, including E-commerce, seem to be examples characterized by the high possibility for game-based learning, as customers can be focused forward into financial increasing efficiency. Due to E-commerce, the cash-less economy has come into existence.

E-commerce is a widely accepted business nowadays, but still, it is taking time to be accepted by all human beings. With each coming day, the ease in the business of E-commerce is expanding at a higher rate (Kotha et al., 2004; Vakulenko et al., 2019). Given the wide range of human differences (Bai et al., 2021; Huang et al., 2022), it can be challenging to determine what factors work the best and which will be avoided. It is widely accepted in the field of E-commerce that intention is a reliable predictor of behavioral findings and a proxy for future purchasing behaviors (Chen and Yang, 2021; Xiang et al., 2022), despite being extremely difficult to quantify. A variety of factors influence the likelihood of making an online purchase. There are many different influencing factors that influence both online and offline purchase intention in different ways and to different degrees. Customer demands, power, and utilitarianism are common characteristics of online consumers, and these characteristics are important distinctions between online and offline consumption. Furthermore, consumers’ lack of leisure time and lifestyle can influence their intention to purchase online (Shao et al., 2021; Qiu et al., 2022; Wang et al., 2022).

There have been a lot of studies performed in the field of consumer habits to develop theories based on the concept of intention. According to Oliver’s expectation and disconfirmation theory (EDT), consumer satisfaction is a function of expectations and disconfirmation of expectations. Satisfaction is thought to have an impact on people’s attitudes and their willingness to buy. The theory of reasoned action (TRA) was developed by Oliveira et al. (2017), and it asserts that persons’ quality is measured by their performance expectancy, which is ascertained by the person’s subjective norms. In addition to product uncertainty in E-commerce, we asserted that consumers’ trust in broadcasters can directly impact their perceived intention (PI). Trust can be recognized as a vital antecedent of faith in online transactions in E-commerce, creating a positive attitude toward transaction behavior (Nasiri and Shokouhyar, 2021), which led to purchase intentions. Previous research has shown that trust is linked to purchase intentions (Paul and Rosenbaum, 2020). Li et al. (2020) discovered that consumers’ intentions to engage in a purchase are influenced by their integrity, while one’s ability impacts their intentions to ask questions about the good or service without making a purchase. There is a positive relationship between purchase intention and actual purchasing behavior (Kumar and Ayodeji, 2021). The consumer’s intention to purchase through E-commerce is defined as PI in this study (Salari et al., 2021). PI is a direct predictor of actual purchase behaviors (Truong et al., 2020). Product lack of certainty (i.e., product fit and top-notch uncertainty) is among the essential functional factors that online shoppers take into account during purchase decisions.

Moreover, customer PI depends on transparent information circulation. Any information gap between customers, vendors, and stakeholders misleads the customers and ultimately affects the business of E-commerce (Kolotylo-Kulkarni et al., 2021). Although customers show concerns at the disclosure of secret information, most of the customers are now getting addicted to E-commerce and do not express any type of reservations. During the COVID-19 pandemic, E-commerce has gained a large share of the market (Pantano et al., 2020). At the time of scarcity, customers have fewer options to select (Hamilton et al., 2019); that is why all the customers ignored their reservations and just used E-commerce to fulfill their needs. As culture also affects the intention of the customer, in China, Korean cultural product perception is better, so they purchase across the border through an E-commerce channel (Han and Kim, 2019). E-commerce is directly related to trust, the same as other offline businesses. The trust comes from consumers’ confidence and particularly awareness of the product. Product awareness comes from more promotion on social and multimedia and when a product has more users in the market. Product awareness may directly affect the intention of the consumers of E-commerce in China. According to Chen and Yang (2021), customer engagement in the system creates intentions in the customer’s mind, and customer psychological factor also improves the intention of E-commerce customers in china.

In China, the E-commerce business is spreading quickly. Alibaba and Tencent have been working in E-commerce at the retail and wholesale levels. These companies have set a positive intention in the mind of customers. With each passing day, the perception of online shopping is changing in China, although China’s economy is already mostly cashless. This type of business works in the presence of thirrd party involvement such as money market funds (MMFs), especially in China (Wang and Ben, 2021). These markets have set a system of financial trust and changed the intention of customers. This system of MMF is not only facilitating financial services but also the point of investment for investors around the globe. The maturity of the payment system has changed the PIs of China’s E-commerce. In this study, we can take Pinduoduo as an example.^1^ This company was established in 2015 and now has more than 824 million users in China. This change has come due to technology acceptance. WeChat has changed the perception, intention, usefulness, and ease of use in China. Besides, this app has shifted the cash economy to a cashless economy (Zhao et al., 2019). WeChat is the first high-ranked payment system globally, and Ali Pay is ranked at the second number (Tran, 2021). In China, the online business system is growing faster, such as Taobao, JD, and Tmall. In the case of grocery retailing, the Chinese market is developing (Olsson et al., 2021), and still, there is the problem of delivery of products while customer perception is good, but the delivery cost and the bottleneck of extra cost are creating problems. According to Geng and Li (2020), two main elements affect the E-commerce intention in China. These are (i) aggressive analysis and (ii) the digitalization of each system. The factorial analysis model depends on these two factors for the E-commerce analysis of China. According to Shan et al. (2020), E-commerce in China is positively associated with the market design and technical performance (Tang et al., 2022). Therefore, the intention-based determinants of E-commerce in different parts of China are perception, availability, usefulness, innovation, technology, urbanization, and technology (Vasic et al., 2019).

The establishment of the E-commerce markets at a bigger rate has damaged offline businesses. All the businesses of whatever criteria, either goods or services, should work on E-commerce. If they ignore the E-commerce concept, they will lose their organizations in the near future. E-commerce in China and around the globe is a matter of serious concern (Xiao et al., 2019). In most of the research, the center of focus is the domestic E-commerce business, but Yoon and Zhang (2018) have worked on the cross-border E-commerce business between China and the world, and it was noticed that E-commerce had changed the intentions of customers not only in China but also in the world.

When the proposed novel factors are combined with the existing factors, this study provides a comprehensive analysis of the intention-based critical determinants of E-commerce utilization in China, according to the findings. Finally, in terms of the significance of the findings, despite the fact that the research was conducted in a specific region of China, the implications of the findings suggest that consumers’ intention factors to use E-commerce are prevalent. E-commerce has huge research potential in China, and the prospect of E-commerce in China is very good. Social commerce, a new E-commerce model, has a significant impact on consumer behavior. By combining information, experience, and social knowledge, consumers can improve their understanding of online PI. As a result, purchasing decisions on E-commerce platforms will be more precise and intelligent. Even though E-commerce is becoming more popular, it is still in its early stages, and only a few social commerce vendors have made a significant profit from it. Other developing economies face the same E-commerce challenges and proposed factors. As a result, the results of this study are generalizable to other economies and demonstrate the influence of intention-based critical factors on the use of e-commerce. Then, we will apply what we have learned from China in order to forecast where this trend is headed. As a result, the findings will assist the Chinese government in determining end users’ intention to use E-commerce.

The theoretical approach is described in the “Theoretical Background” section, followed by the “Materials and Methods” section, in which we proposed a research model of the intention-based critical determinants of E-commerce utilization. We first described how our evidence-based study was carried out and then revealed the study’s findings (segment 4). The discussion and conclusion are presented in the “Results” and “Discussion” sections, respectively.

## Theoretical Background

Technology Adaptation Theory (TAT) presents the intention and behavior of an individual toward the acceptance of technology. E-commerce is derived from technology. This theory consists of two factors: the result of perceived value and a person’s behavioral change due to his/her belief and motivation. According to Bijmolt et al. (2010), E-commerce learning comes from three steps. The first step leads toward the attraction of new customers in second phase, the customer development. In the second stage, the repetitive customer repurchase starts. In the final step, we came to know the loyalty of the customers. According to Gilboa et al. (2019), customers who are regular and loyal to the company are not like ordinary customers in E-commerce. The intentions of a loyal customer are different from others. Nowadays, organizations are working to make their loyal E-commerce customers by delivering batter (Vasic et al., 2019). According to Lowery (2021), the trust of customers in E-commerce changes their intention. It depends on stakeholders’ activities, better image of the web content, customers’ simplicity of using the online platform, and customer firm belief regarding particular retailers. E-commerce trust depends on the elements such as courage, benefits, and skills (Kim and Gupta, 2009). Mental accounting theory expresses the stages of E-commerce transaction, in the first stage, it evaluates the transaction, and in the second stage, it takes the final decision (Kim and Gupta, 2009). After these two-step customers with absolute thinking, the organizational performance of specific E-commerce businesses is assessed (Hamilton et al., 2019).

Transaction in E-commerce has greater importance because many companies or some intermediates do fraud with the end customer (Keshri et al., 2020). Frauds change the intention of customers in E-commerce. According to Kolotylo-Kulkarni et al. (2021), information processing theory gives a choice to the customer in his decision-making process than he takes the decisions at the past E-commerce experience. Past customer experience has an impact on the perception and intention of E-commerce. In previous studies, it has been known that the E-commerce repurchase ratio is very low, and 0.50% of customers do not visit the site again. According to Leopoldo (2019), E-commerce also depends on mobile and the Internet, which develops the infrastructure of E-commerce. E-commerce in the cities is growing much as compared with rural areas, and it is due to facilities of Internet and knowledge gap. According to Cheba et al. (2021), determinants of E-commerce in China are the availability of mobile and Internet, country macroeconomics situation, social condition, environmental performance, and E-commerce business in cities. All these factors affect the E-commerce consumer’s intentional behavior in China and around the globe. In previous research, different aspects have been covered but in this research, the purpose was to judge the impact of intention-based perception, usefulness, reputation, ease of use, belief in vendor, and purchase frequency by E-commerce in China concerning the end customer. The research framework for this study is depicted in Figure 1.

**FIGURE 1:** Research framework.

### Perceived Usefulness in E-Commerce

Consumers’ general preconceptions of the risks and benefits associated with a customer experience are regarded as perceived values. Beyond the straightforward impact of perceived usefulness (PUSF) on implementation, research has found that PUSF can act as a mediator in a variety of disciplines. Similarly, PUSF has been found to establish a relation between perceptual customization and buying intention in E-commerce (Feng et al., 2021). That is, greater cognitive behavior, or the intensity to which users are satisfied with the information, is given in a specific product and is linked to higher repurchase intention for such a good or service. This connection exists due to the mediating effects of the consumer’s perceived usefulness (Kim et al., 2021). The study explains to the E-commerce consumers how ready and able to use the Internet to purchase goods. Another thing related to customer consent is sharing personal information with invisible representatives. The customer consent to cooperate with a web-based E-commerce system directly linked with the usefulness of the system. In E-commerce, the website’s front page is where potential customers can find out more about the company’s services and expertise (Kim et al., 2021). In general, it is a very simple system, and in the advanced concept of organizations, it is a multidimensional system and very complex (Hopkins, 2022; Kliestik et al., 2022b). Another important aspect examined in this study is the degree of use and repetitive visiting site behavior, which is due to the usefulness perception and their collaboration to share personal and Internet-based data (Nica et al., 2022). Online interactions such as ease of information collection, updated information, and entertainment are not only the choices, which are essential for making a decision but they also create an image with the help of the first website attempt and observations. So, E-commerce is the formative behavior that comes from continuous, repetitive Internet-based activities.

*H_1_: Perceived usefulness has a positive impact on consumer’s intention to use E-commerce systems.*

### Perceived Ease of Use in E-Commerce

Perceived ease of use in E-commerce is outlined as “the degree to which the person believes that exploitation the system new school are going to be freelance of brainpower” (Kasilingam, 2020). This ease of handling the results with an ideal mindset conveys the idea. Reports tailored to a person’s locus of control, in specific, take place effortlessly to digest. Likewise, Zhang et al. (2020) discovered that a mark promotional material corresponding to a regulative objective looks easier to perform than one that does not. This same easiness of its use had also piqued the interest of researchers interested in areas other than ancient production and design development. In general, a practical amount of physical and mental effort is necessary to know, learn, and operate a specific technological system (Kliestik et al., 2022a). Ease of use may be defined in the way that buyer’s discernment of a by-product, notably in any way commodity is simple to absorb and utilize, shrinks the weight of remembrance, and provides a high level of satisfaction. The ease of use of software, or the transparency of work and easy way finding, is a compulsory situation for E-commerce selling to get through and set off with success (Ashraf et al., 2021).

This quality concerns buyers’ online shopping etiquette structure. Furthermore, customers will shift their attention to other apps whenever the person’s laptop relation to software is not sufficiently affectionate to boost their sales. Thus, assessing the usability of software in E-commerce selling is required. The usability of mobile applications is not enough to determine consumer behavior. It is also an essential element for product developers looking to improve device design. As a result, when consumers come across different mobile applications from E-commerce businesses, they should choose the one with the greatest easiness of its use.

*H_2_: Perceived ease of use has a positive impact on consumer’s intention to use E-commerce systems*

### Reputation in E-Commerce

Seeing as the rumor mill can negatively impact the reputation of an E-commerce business, the thousand-dollar concern is to save virtual customers’ beliefs in E-commerce and its Internet-based financial activities. Therefore, rumor-based consumers are divided into four categories, namely, online customers, puzzled customers, customer left, and rebuying consumers (Bellini et al., 2020). It is well known that E-commerce consumers face several challenges such as fraudulent selling, quality issue, bad services, and risk factors that affect the reputation of the E-commerce business (Vãtãmãnescu et al., 2020; Andronie et al., 2021). To address these issues, famous E-commerce enterprises such as https://productsearch.alibaba.com/, Walmart, JD, and Taobao frequently and broadly enforce reputation systems (Zhao et al., 2020). A repetitive buyer is someone who buys from the same vendor a second time, and on a daily basis, the repetitive customers spend more and more money (Kolotylo-Kulkarni et al., 2021). Buyback conduct impacts repeat intention activities, and it also shows the trustful relationship between consumers and retailers. It should be focused on when setting seller reputation and purchaser demand (Kasilingam, 2020).

According to Bellini et al. (2020), there are many fake comments and ratings on the popular retailing platform. As a result, consumers may be misled by these fake comments and ratings while online shopping. This type of abnormal rating is known as a malicious rating, and those who give malicious ratings have been known as attackers. These types of malicious can be detected by analyzing the previous rating, and many approaches have been unveiled to detect these attackers (e.g., Ashraf et al., 2021). This reputation may impact the future decision-making of consumers. When there are no nefarious scores, the product reputation can be maintained. To manage these types of fatal attacks, the 3R (repurchase, return, reputation) model has been discovered by researchers.

*H_3_: Reputation of websites used by vendors has a positive impact on consumer’s intention to use E-commerce systems.*

### Trust in Vendors in E-Commerce

In an E-commerce environment, trust is both important and vulnerable (McKnight et al., 2002). Consumers’ perception and uncertainty could be reduced by trust. To predict the issues in vendor trust, the customer service life cycle is used in many types of research (Kolotylo-Kulkarni et al., 2021). It consisted of the whole set of the system from collecting the information about any product, purchasing it, disposing, and even replenishing it (Zhou et al., 2018). It also reduces the state of mistrust between vendors and customers and gives a transparent purchasing system. The buyer-perceived system of transparency is the set of three elements that could be transparent: vendor, product, and transaction detail. According to Ribadu and Wan (2019), many customers do not believe in E-commerce; it negatively influences buyers during purchasing through the Internet. Consumer trust, vendor’s reputation in the market, and quality assurance are the main elements that impact E-commerce.

As a result, there is very difficult to establish or maintain trust between vendor and consumer in E-commerce. The E-commerce literature defines consumer trust in e-suppliers as a positive psychological state, based on beliefs in professional knowledge (Kasilingam, 2020), integrity, and generosity to determine the tendency to participate in trust-related behaviors (Cui et al., 2018). Online trust has been classified into four categories: trust based on the first impression, trust based on regular contact, trust on personal characteristics, which finally lead to the success just on a company’s market picture.

*H_4_: Trust in vendors has a positive impact on consumer’s intention to use E-commerce systems*

### Purchase Frequency in E-Commerce

Purchase frequency is the range of times a client makes a sale in a very given amount of time (Ingham et al., 2015). Further buying rhythm explores the image in the mind of customers that influence consumers to buy through the Internet, even while observing the mediating impact of e-buying expertise. McKnight et al. (2002) differentiate two types of attitudes: acceptance of E-commerce is the first repurchase of goods and buying back and behavioral intention is the repeating behavior of repurchase using the same medium. Yu et al. (2005) claimed that new possible customers of an E-commerce differ from repeat usage in order of acceptance, intentions, and usage. The same occurrence is explained by Oliver (1980)’s Expectation-Confirmation theory. It appears perfectly reasonable to believe that large acceptance ends up with a large frequency of use and, as a result, larger satisfaction. According to Le et al. (2021), the most powerful generator of self-efficacy influences because the skills acquired through Internet use determine this perception. Recurrent Internet users should be more identity and thus more likely to benefit from E-commerce. We can consider the buyers who have more steering professionalism, which connects to the Internet more frequently, are comfortable with it, and have a greater self-efficiency in E-commerce.

*H_5_: Purchase frequency has a positive impact on consumer’s intention to use E-commerce systems*

## Materials and Methods

### Questionnaire Development

The study method was verified quantitatively using a rating scale that had earlier been proven to work to actualize each structure and boost its authenticity. As a result, in the advancement of measurement devices, this was adjusted from validated empirical investigations. We then designed a questionnaire to achieve the study purpose. The very first portion of the questionnaire comprised specimen classification questions. The second section evaluated the structures chosen using a seven-point rating scale (1-strongly disagree, 7-strongly agree). As per the literary works, in IS, common method bias (CMB) is a major worry about data gathering operational definition. We calculated the Harman feature to evaluate CMB, and all predictors were allowed to pass that check (less than 0.5) (Schwarz et al., 2017). The final tools of measurement often used to check the structural model are listed in Appendix A. To make sure a widely accepted set of questions, the survey was performed using established balances. Participants were asked about single-game element key findings (Huang et al., 2020), so they were not anticipated to have previous information on game element design systems.

**TABLE 1:** Participants’ demography.

Sample characteristics	Frequency	Percentage *n* = 400 (%)
**Gender**		
Female	164	41.00
Male	236	59.00
**Age**		
<25	67	16.75
25–35	198	49.50
35–40	97	24.25
>40	38	9.50
**Education level**		
High School	55	26.96
Bachelor	84	41.18
Post Graduate studies	23	11.27
Master	40	19.61
PhD	2	0.98
**Income**		
Less than 10,000 RMB	30	7.50
10,001–15,000	70	17.50
15,001–20,000	105	26.25
20,001–25,000	138	34.50
25,001–30,000	39	9.75
More than 30,000	18	4.50
**Marital status**		
Married	285	71.25
Unmarried	115	28.75
**Occupation**		
Technical personnel	166	41.50
Government job	27	6.75
Own business	115	28.75
Other	92	23.00

### Selection of Respondents and Sample Size

To make certain that their results were accurate and meaningful, the researchers conducted a pilot survey before starting the main study (Xue et al., 2014). Random sampling was used to ensure that all members of the subset had an equal chance of being selected as a part of the sampling process in order to avoid an unbalanced representation of the overall population (Tauni et al., 2015). The survey process was divided into two phases. First, questionnaires were handed over to 500 consensual E-commerce website users in both the business-to-customer (B2C) and customer-to-customer (C2C) contexts, with a high prevalence in the propagation of the survey on social networks. We provided an online survey link to respondents *via* Linkedin, Facebook, and Whatsapp. One month was allotted for the completion of the responses, and they were all completed on time. An in-depth explanation of the questionnaire was given to the participants to ensure that they understood all aspects of the questionnaire. Participants reflected in the following online vendors: AliExpress 13 percent, Amazon 18 percent, Made an impact 3 percent, Continent 1 percent, eBay 20 percent, El Corte Ingles 1 percent, Lot 12 percent, GearBest 8 percent, PCDiga 4 percent, Sporting 2 percent, Worten 4 percent, and on vendors 10 percent. The portrayal of the specimen is outlined in Table 4.

Second, questionnaires were received from the respondents after 1 month. As a result of the questionnaire survey, a total of 400 responses were collected, representing 80% of the original sample. Based on Westland’s sample size calculation formula, the recommended minimum sample size for our model should be 336 (Westland, 2010), while our actual sample size (400 responses) is even more than the minimum recommended value, ensuring that empirical analysis is feasible. Users were asked about the conceptions of their own life experiences with B2C and C2C systems. Besides they were asked about their most utilized E-commerce console, not just one.

### Statistical Analysis

AMOS (edition 26) and SPSS (edition 26) softwares are used for statistical tests. Structural equation modeling (SEM) is used to test the hypotheses. SEM is a practical approach for determining the relationship between various variables, providing meaningful and accurate results (Liu M. et al., 2021), with three significant advantages over traditional methods. (i) An accurate assessment of measurement errors. (ii) Using identified variables to approximate underlying features. (iii) Tool for modeling for trend evaluation and implementation based on data compliance. Furthermore, most multinomial strategies tacitly dismiss math errors. The SEM, on either hand, forecasts both variables of the study while accounting for miscalculation (Sardeshmukh and Vandenberg, 2013). The method creates precise and erudite numbers due to its reliability and serviceability.

The SEM method enables the generation of various predictor structures for every component as well as yields audio ramifications. Furthermore, it calculates the mistakes parts of the work carefully. As a consequence, the connection among variables produces accurate results. Furthermore, this can evaluate complicated interactions as well as a wide range of assumptions by incorporating average setups and team market values, what other designs and experiments could do (Agudo-Peregrina et al., 2014). Taking the benefits of SEM in and out of evaluation, we used it with our assessment because it is the most effective method to test the association between the variables under evaluation.

## Results

### Demography of the Participants

Table 1 presents the demography of the participants. The lower-middle age group (198, 49.50%) has the highest percentage of respondents in our sample, followed by the middle-age group (97, 24.25%), young age group (67, 16.75%), and old age group (38, 9.50%). In our sample, male participants are 236, 59.00% of the whole sample, and outnumbered females 164 (41.00%). With a monthly income of 15,001–20,000 CNY, 185 respondents (26.25%) are from the middle-income class, followed by the upper-middle-income class (198, 39.5%) with a monthly income of 25,001–30,000 CNY. We also divided respondents into groups based on their educational levels; 26.96% have a high school diploma, while 41.18% only have a Bachelor’s degree. The majority of the respondents were married (71.25%), 41.50% are technical persons, and 6.75% worked for the government.

### Descriptive Analysis and Correlation Analysis

The hypotheses were tested after the initial screening of responses for usability and reliability (see Table 2). The data in this study were analyzed in two steps. For the model’s validity, we conducted a confirmatory factor analysis (CFA). The proposed research model’s causal structure was tested using structural equation modeling (SEM). Modifying the proposed model using the model-generating (MG) strategy for testing structural equation models was carried out until it met the criteria for theoretical significance and statistical well-fitting (Jöreskog, 1993). The formative and reflective latent variables were measured during the evaluation of the measurement model. Tests of indicator reliability, internal consistency, discriminant validity, and convergent validity were used to evaluate the reflective latent variables’ measurement model (see Table 3). When factor loadings for perceived desirability were examined for indicator reliability, some poor factor loadings were discovered. These items were omitted from consideration for this study. When the test was rerun, the factor loadings for all remaining reflective indicators were found to be greater than or equal to the 0.70 threshold, which was deemed acceptable. To test the construct’s validity, data variance was compared for both discriminant and convergent validity, and both were found to be statistically significant. Table 4 shows that all constructs are significantly higher than the threshold of 0.50. Convergent validity testing necessitates factor loadings and average variance extracted (AVE) of all constructs to be at least 0.50. In addition, correlations between each construct and every other construct were smaller than the square root of the AVE of each one, as shown in Table 4, for discriminant validity using the Fornell and Larcker’s (1981) criterion.

**TABLE 2:** Results of descriptive statistics.

Variables	Items	Observations	Coefficient of variation (CV)	Mean	Std. Dev
PUSF	5	400	0.147	3.731	0.518
PEUS	4	400	0.588	2.863	1.588
REPU	4	400	0.081	3.406	0.258
TVEN	7	400	0.129	4.036	0.493
PFRE	6	400	0.225	2.748	0.583
IUES	4	400	0.605	3.069	1.751

*PUSF, straightforward impact of perceived usefulness; PEUS, perceived ease of use; REPU, reputation; TVEN, trust in vendor; PFRE, purchase frequency; IUES, intention to use E-commerce systems.*

**TABLE 3:** Correlation and discriminant validity analysis.

Variables	PUSF	PEUS	REPU	TVEN	PFRE	IUES	AVE	MSV
PUSF	(0.715)						0.512	0.122
PEUS	0.267	(0.821)					0.674	0.292
REPU	0.349	0.540	(0.802)				0.643	0.292
TVEN	0.304	0.160	0.352	(0.844)			0.712	0.124
PFRE	0.155	0.354	0.259	0.227	(0.824)		0.678	0.445
IUES	0.284	0.493	0.429	0.216	0.667	(0.744)	0.554	0.445

*Diagonal values in parentheses represent the root square of average variance extracted (AVEs).*

**TABLE 4:** The results of reliability analysis and factor loadings.

Variables	Items	Standard loadings	Cronbach-α	CR
Perceived usefulness			0.813	0.807
	PUSF 1	0.737		
	PUSF 2	0.802		
	PUSF 3	0.920		
	PUSF 4	0.866		
	PUSF 5	0.880		
Perceived ease of use			0.916	0.935
	PEUS 1	0.719		
	PEUS 2	0.731		
	PEUS 3	0.731		
	PEUS 4	0.675		
Reputation			0.910	0.915
	REPU 1	0.880		
	REPU 2	0.959		
	REPU 3	0.709		
	REPU 4	0.695		
Trust in vendor			0.903	0.925
	TVEN 1	0.634		
	TVEN 2	0.841		
	TVEN 3	0.802		
	TVEN 4	0.869		
	TVEN 5	0.833		
	TVEN 6	0.835		
	TVEN 7	0.893		
Purchase frequency			0.832	0.893
	PFRE 1	0.851		
	PFRE 2	0.736		
	PFRE 3	0.661		
	PFRE 4	0.914		
	PFRE 5	0.907		
	PFRE 6	0.657		
Intention to use E-commerce systems			0.809	0.832
	IUES 1	0.746		
	IUES 2	0.710		
	IUES 3	0.762		
	IUES 4	0.609		

*Rotation method: Promax with Kaiser normalization and extraction method: maximum likelihood.*

### Reliability Analysis

Cronbach’s alpha was computed to assess the reliability coefficient. The findings demonstrate that the Cronbach’s value for all factors exceeded the lowest required value of 0.70, as recommended by Treiblmaier and Sillaber (2021), verifying the data’s accuracy. It was decided to use composite reliability (CR) assessment to see if all the explanatory variables were consistent. CR values are found to be higher than the recommended threshold of 0.70, as determined by the investigation (Hair et al., 2017). Table 4 presents the conclusion.

### Multicollinearity

To test the multicollinearity, regression was used to determine the value systems of the variance inflation factor (VIF) as well as tolerance. As per the *f*, the value of VIF has to be less than 10, and the tolerance value has to be larger than 0.1. The research results indicate that the model did not have a multicollinearity problem, so the VIF value is as per limit, and the value of tolerance for whole variables ranges within the ideal range and is in line with the observations of Strupeit and Palm (2016). The findings can be seen in Table 5.

**TABLE 5:** The results of the collinearity diagnostic test.

		
Variables	Statistics for collineraity	
	Tolerance	VIF
PUSF	0.853	1.172
PEUS	0.937	1.067
REPU	0.801	1.248
TVEN	0.836	1.196
PFRE	0.946	1.057

*Dependent variable: IUES.*

### Factor Analysis

To acquire the attributing design methodology, an exploratory factor analysis (EFA) has been conducted. EFA seeks to explore factorability, i.e., the relationships and clusters of different factors based on cross-comparisons (Mahmood et al., 2019). For even more meaningful results, the factors were derived to use the statistical parameters and then turned with the corresponding Varimax coefficients. The Eigenvectors have been used to assist specify the number of factors. Several tests that were carried out during this stage are crucial to determine whether the EFA might be applied in this study. The Bartlett’s Test of Sphericity (BTS) and Kaiser-Meyer-Olkin (KMO) test were used to evaluate the data fitness. The consequences supplied a significance based on KMO (Kaiser, 1974), implying that principal component analysis can be continued. Table 6 presents the results of the KMO and BTS tests. The substantial significance of 6,874.96 provided by BTS also meets the requirements for EFA. Table 7 results show that almost all factors have a value greater than the standard minimum of 0.4, consequently (Stevens and Stevens, 2001). There are seven important factors that have Eigenvalues larger than one and a total combined variability of 64.930% for the Promax roster using the Kaiser method (Table 8). Since each one of these is true, the data can be trusted to support further assessment (Blunch, 2017).

**TABLE 6:** Bartlett’s test and Kaiser–Meyer–Olkin (KMO).

KMO and Bartlett’s test		
Kaiser-Meyer-Olkin Measure of Sampling Adequacy		0.908
Bartlett’s Test of Sphericity	Approx. Chi-Square	6,874.96
	df	435
	Sig.	0.000

*Sig, significance, df, degree of freedom.*

**TABLE 7:** Communality findings.

Variables	Communalities	
	Initial	Extraction
PUSF	1.00	0.544
PEUS	1.00	0.679
REPU	1.00	0.918
TVEN	1.00	0.575
PFRE	1.00	0.630
IUES	1.00	0.768

*Maximum likelihood: extraction method.*

**TABLE 8:** Cumulative variance and Eigenvalues.

Variables	Eigenvalues (initial)			Squared loadings extraction sums		
	Total	Variance%	% Cumulative	Total	Variance%	% Cumulative
1	9.669	32.229	32.229	9.280	30.935	30.935
2	3.746	12.487	44.716	3.418	11.394	42.329
3	3.000	10.000	54.715	2.635	8.784	51.114
4	2.083	6.942	61.658	1.695	5.650	56.764
5	1.983	6.611	68.269	1.650	5.499	62.263
6	1.141	3.804	72.073	0.800	2.667	64.930

*Rotation method: cumulative variance, Promax with Kaiser normalization: 64.930%.*

Later, the models were discovered *via* confirmatory factor analysis (CFA). CFA can be used to verify the EFA framework of variables. Finding out if a model is normal is the first step in making a model selection. Items with high capacities (greater than 0.7) should always be available (Truong et al., 2020). According to the findings, all levels were found to be greater than 0.7. Since all goods were packed on one’s own constructs, the validity of the quantification model was confirmed (Figure 2). Data can be reused in the measurement model following the completion of the analysis.

**FIGURE 2:** Confirmatory factor analysis is a type of statistical analysis that is used to represent a measurement model. Source: Authors’ calculations.

### Hypothesis Results and Structural Model

The writers evaluated the proposed prototype and theorized interconnections within a week of acquiring valid and reliable measures. To determine how much variation in the dependent variable could be explained by variation in the independent variable, *R*^2^ was a critical step. The value of *R*^2^ was 0.54, and the difference between the two levels is greater than the corresponding minimal level of 0.35 (Huang et al., 2020), suggesting an important viewpoint. To investigate the model’s connections, we used structural bend assessment and the SEM method. The assessment created a high *f*-value, implying that all interconnections were straightforward. Various fit indices were also used to confirm that the data are accurate and completely fit again for the structural equation model. The results indicate that almost all fit indices (i.e., CFI = 0.988, NFI = 0.923, IFI = 0.989, TLI = 0.974, GFI = 0.983, RMSEA = 0.021, *X*^2^/df = 1.147, and SRMR = 0.026) meet the standard criteria, indicating that model fit the data adequately (Lucianetti et al., 2018).

Figure 3 depicts a diagrammatic diagram of SEM together with path coefficients. The path coefficients for the variables “perceived usefulness,” “perceived ease of use,” “reputation,” “trust in vendor,” and “purchase frequency” H1 (*b* = 0.04, *p* = 0.001), H2 (*b* = 0.13, *p* = 0.01), H3 (*b* = 0.67, *p* = 0.05), H4 (*b* = 0.02, *p* = 0.001), and H5 (*b* = 0.16, *p* = 0.05) demonstrate that the factors PUSF, PEUS, REPU, TVEN, and PFRE have a positive and significant effect on customers’ intention to adopt E-commerce. As a result, assumptions 1, 2, 3, 4, and 5 were acknowledged. Table 9 depicts the authenticity of theorized routes and theories.

**FIGURE 3:** Structural equation modeling path diagram. Insignificant and significant paths are indicated by dashed and continuous lines, respectively. ^***^p < 0.00, ^**^p < 0.01, *p < 0.05. Source: Authors calculation.

**TABLE 9:** Result hypothesis testing.

Hypotheses	Structural paths	β-value	*f*-value	Result	*R* ^2^
H1	PUSF → IUES	0.04***	193.3***	Accepted	0.54
H2	PEUS → IUES	0.13**	145.3**	Accepted	
H3	REPU → IUES	0.67*	108.2*	Accepted	
H4	TVEN → IUES	0.02***	202.8***	Accepted	
H5	PFRE → IUES	0.16*	207.2*	Accepted	

***p < 0.00, **p < 0.01, *p < 0.05.

### Testing Endogeneity

This test is mainly used to verify the consistency of study findings. Endogeneity partiality in the information can jeopardize the findings. Furthermore, endogeneity could misrepresent the forecast of posterior probability, presenting a major challenging problem to the authenticity of outcomes. While investigating endogeneity, we used the Heckman test to address these issues. The results produced the very same degree of confidence as the original version, implying that endogeneity partiality is just not prevalent in our conclusion (Table 10).

**TABLE 10:** Test for endogeneity.

Hypotheses	Structural paths	β-value	*t*-statistics
H_1	PUSF → IUES	0.132***	2.953
H_2	PEUS → IUES	0.354	8.702
H_3	REPU → IUES	0.471***	2.171
H_4	TVEN → IUES	0.383***	3.265
H_5	PFRE → IUES	0.186**	6.761

***p < 0.00, **p < 0.01, *p < 0.05.

## Discussion

This study accomplishes two significant impacts. First, it recommends a conceptual model that combines technology adoption theory with the implication of the E-commerce system of business. As a result, incorporating aspects of adoption studies, combined with E-commerce models, including facets of much other research. Second, we evaluated this study model in terms of actual E-commerce platform utilization. As a consequence of our research, customer E-commerce platform implementation is straightly attributable to the concentration of perceived usefulness, perceived ease of use, reputation, trust in vendor, and purchase frequency, which also produce a customer sense of giving rewards as a result. The study’s findings are consistent with the literature, namely, the Technology Adoption Theory (Venkatesh and Davis, 2000).

### Perceived Ease of Use

The results show that perceived ease of use and perceived usefulness have a significant positive impact on IUES. This finding implied that the more an individual felt capable of using an application, the easier it was for them to use an E-commerce system. This result also implied the ease they felt from using the application, as consumers carried over into their perception of ease they felt toward using the application as a customer or seller. Further development of an E-commerce application that is easy to use increases the number of existing customers in general (Huang et al., 2021) and increases the number of E-commerce partners the application has, thus providing more (Liu P. et al., 2021). This finding was consistent with the previous research that showed the significant positive impact of perceived ease of use (Moorthi et al., 2021) and attitude toward E-commerce intention (Lăzăroiu et al., 2020). Although the perceived usefulness result was inconsistent with the aforementioned extant corpus, some of the previous findings still showed similar results (Spruit and Almenar, 2021; Zheng et al., 2021). This result implied that rather than the usefulness of an application, its easiness and attitude toward it were the variables that determined its adoption. In other words, even if an application was provided to be useful, as long as it was hard to use or ignited a negative attitude, no one would want to use it.

### Perceived Usefulness

Perceived usefulness has a significant positive result on IUES. Consistent with previous research, perceived usefulness plays an important role in defining the intention of using E-commerce systems (Liu X. et al., 2021; Yang et al., 2022). The usefulness of an application depends on its ease of use (Cremer and Loebbecke, 2021). The previous statement implied that, for individuals, an application would only feel useful when it is easy to use (Yuan et al., 2021). This also means that for application developers to ensure that their application is useful to users, they need to consider the application’s ease of use. Consumer shopping experiences are being improved, and retailers are remaining competitive by implementing E-commerce (Sharma and Aggarwal, 2019). Consumers’ purchasing experiences were examined by Chen and Yang (2021), who studied the impact of mobile retailing. The findings of this study can help other researchers better understand how technology usefulness affects consumer behavior, emphasizing the factors that motivate consumers to adopt the e-commerce shopping experience. Customers’ perceptions of the attributes of e-commerce that influence their cognitive and affective attitudes and online purchase intentions were studied by Ribadu and Wan (2019). Utilitarian attributes are found to be a significant and positive predictor of cognitive and affective attitudes, according to the authors.

### Reputation

Furthermore, reputation has a significant positive impact on IUES. Reputation is generally considered to be an important factor in long-term customer relationships and customer trust. Previous research (Akram et al., 2021; Aparicio et al., 2021) has found that perceived reputation significantly impacts online shopping trust and purchase intention. A company’s reputation is built on long-term investments of resources (Karani and Failler, 2020), effort, and attention (Meilatinova, 2021) to customer relationship building. Consumers prefer companies with a good reputation in E-commerce because they perceive less risk and uncertainty and are aware of where to seek assistance. These findings are consistent with theory and prior studies (Qalati et al., 2021).

### Trust in Vendor

The hypothesis that IUES is significantly affected by trust in vendor-related hypotheses (F2 > 0.383) and is highly significant (*p* < 0.000) is supported by the data. The results of the SEM model show that online trust occurs in E-commerce and that trust has a major impact on satisfaction and repeat purchase intention. The value is higher than in prior E-commerce research investigations (Aparicio et al., 2021). In the e-commerce context, trust is a crucial aspect to investigate: many small and medium online sellers do not aim to use their website as a channel since there are numerous obstacles (Qalati et al., 2021), such as trust concerns when doing business at a distance and uncertainties, and increased risks. Moreover, if customers have faith and trust the online vendor that the vendor will be honest and reliable, they will be more likely to feel comfortable making purchases and disclosing sensitive information online (Wang and Emurian, 2005). According to Sharma and Aggarwal (2019), customer happiness can be improved by delivering high-quality products and websites that customers trust. This can be accomplished through delivering a great customer experience and differentiated services, which will lead to positive purchase decisions.

### Purchase Frequency

This analysis revealed interesting insights into how consumers changed their online E-commerce purchasing habits regarding purchase frequency. The frequency shifted evidently toward a substantial and increased E-commerce use (Yu and Huang, 2022), with the population ordering more than once per month increased by 44.5%. In addition, the percentage of people never ordering through online channels decreased by more than 50% (Kawasaki et al., 2022). This is a clear sign that purchase frequency has increased the use of online channels in China, as the statistical tests in the previous section also demonstrated. The test results show that the increase in use will also increase the satisfaction with delivery services (Böheim et al., 2021). This could be due to the fact that the most experienced and loyal users frequently use the most reliable and best online retailers and do not experience any unpleasant surprises when doing so (Gian et al., 2019). The navigated and less loyal consumers may incur bad or unreliable websites, and as a result, they will have a worse shopping experience.

## Conclusion

This study systematically assessed intention-based critical determinants of E-commerce utilization in China. We identified the potential factors that could discourage or inspire consumers from using E-commerce. The conceptual framework of Technology Adaptation Theory (TAT) presents the intention and behavior of an individual toward the acceptance of technology. The theory contains two factors: the result of perceived value and the other is that people’s behavior changes due to beliefs and motivations. SEM/PLS was used to analyze survey data collected from the four largest cities in Guangdong Province. The empirical analysis discloses that perceived usefulness, ease of use, reputation, trust in vendors, and purchase frequency positively influence E-commerce utilization.

Customers purchase the market image and market reputation of E-commerce channels as well. Additional core functions of E-commerce Internet sites, such as making purchases faster and spending less time on unnecessary activities, have a strong positive effect on behavioral intention. The interface and ease of use are also important factors in the E-commerce customer experience. Companies can improve their trustworthiness in the eyes of their customers by ensuring improved quality; fulfilling the given promise enhances the level of commitment, integrity, and level of trust. This exploration has some limits. Initially, data were collected only from E-commerce customers. In terms of age, the reality that even more than 80% of survey participants are aged 30 years or younger, and the fact that more than 87% of the sample chooses to live in Shenzhen and Guangzhou may impact the outcome acquired. Even though the research results seem to be statically meaningful, so much study with a wider geographical purview will improve the model’s predictive power.

## Data Availability Statement

The raw data supporting the conclusions of this article will be made available by the authors, without undue reservation.

## Ethics statement

The studies involving human participants were approved by the Ethical Committee and responsible authorities of Henan Agricultural University following all guidelines, regulations, legal, and ethical standards as required for humans. The patients/participants provided their written informed consent to participate in this study.

## Author Contributions

Both authors listed have made a substantial, direct, and intellectual contribution to the work, and approved it for publication.

## Conflict of Interest

The authors declare that the research was conducted in the absence of any commercial or financial relationships that could be construed as a potential conflict of interest.

## Publisher’s Note

All claims expressed in this article are solely those of the authors and do not necessarily represent those of their affiliated organizations, or those of the publisher, the editors and the reviewers. Any product that may be evaluated in this article, or claim that may be made by its manufacturer, is not guaranteed or endorsed by the publisher.

## Footnotes

1
https://en.pinduoduo.com/

## Appendix

**Appendix A:** Survey questionnaire.

Constructs	Items	Strongly disagree	2	3	4	Strongly agree
**Perceived usefulness**						
PUSF 1	E-commerce websites provides an interface that tracks the delivery status of purchased products/services					
PUSF 2	E-commerce websites provides an interface that efficiently handles queries of the customers					
PUSF 3	E-commerce websites provides various payment options					
PUSF 4	E-commerce websites provides an interface through which customers can compare the prices of products/services from multiple vendors					
PUSF 5	E-commerce websites provides an interface with significant content about products/services					
**Perceived ease of use**						
PEUS 1	E-commerce websites provides an interface with smooth payment process					
PEUS 2	E-commerce websites provides the customers an opportunity to build their own shopping carts.					
PEUS 3	E-commerce websites offer complimentary products/services according to recent search					
PEUS 4	E-commerce websites provides an interface that posts linguistic comments provided by previous purchasers and browsers.					
**Reputation**						
REPU 1	I am satisfied with the E-commerce websites					
REPU 2	I will again make a purchase from the E-commerce websites					
REPU 3	The performance of E-commerce websites meet my expectations					
REPU 4	I feel easy to complete the transaction on the E-commerce websites					
**Trust in vendor**						
TVEN 1	I feel safe while sending my personal information to the E-commerce websites					
TVEN 2	E-commerce websites provides exact information about the products/services without any discrepancies					
TVEN 3	E-commerce websites assure the customers that there is no breach of personal information while making a transaction					
TVEN 4	E-commerce websites keep customers’ personal information confidential and protect their data from being included into their database which may be used for any other purpose apart from the purpose it was meant for					
TVEN 5	Purchasing on the E-commerce websites will not cause financial risk					
TVEN 6	The electronic payment on the E-commerce websites is safe					
TVEN 7	The E-commerce websites only collects users’ personal data that are necessary for its activity					
**Intention to use E-commerce systems**						
IUES 1	I am willing to use E-commerece system because I have knowledge about it					
IUES 2	I am willing to use E-commerece system due to its time-saving behavior					
IUES 3	I am willing to spend more on E-commerece system compared to conventional offline systems					
IUES 4	I am willing to use E-commerece system due to its secure nature					
